The article "The Role of the Stem-Loop A RNA Promoter in Flavivirus Replication" was published in 2021. Journal: Viruses.

# The Role of the Stem-Loop A RNA Promoter in Flavivirus Replication

**DOI:** 10.3390/v13061107

**Published:** 2021-06-09

**Authors:** Kyung H. Choi

**Affiliations:** Department of Biochemistry and Molecular Biology, Sealy Center for Structural Biology and Molecular Biophysics, The University of Texas Medical Branch, 301 University Boulevard, Galveston, TX 77555, USA; kychoi@utmb.edu

**Keywords:** viral RNA promoter, stem-loop A (SLA), flavivirus, Dengue virus, Zika virus, polymerase NS5, viral replication

## Abstract

An essential challenge in the lifecycle of RNA viruses is identifying and replicating the viral genome amongst all the RNAs present in the host cell cytoplasm. Yet, how the viral polymerase selectively recognizes and copies the viral RNA genome is poorly understood. In flaviviruses, the 5′-end of the viral RNA genome contains a 70 nucleotide-long stem-loop, called stem-loop A (SLA), which functions as a promoter for genome replication. During replication, flaviviral polymerase NS5 specifically recognizes SLA to both initiate viral RNA synthesis and to methylate the 5′ guanine cap of the nascent RNA. While the sequences of this region vary between different flaviviruses, the three-way junction arrangement of secondary structures is conserved in SLA, suggesting that viruses recognize a common structural feature to replicate the viral genome rather than a particular sequence. To better understand the molecular basis of genome recognition by flaviviruses, we recently determined the crystal structures of flavivirus SLAs from dengue virus (DENV) and Zika virus (ZIKV). In this review, I will provide an overview of (1) flaviviral genome replication; (2) structures of viral SLA promoters and NS5 polymerases; and (3) and describe our current model of how NS5 polymerases specifically recognize the SLA at the 5′ terminus of the viral genome to initiate RNA synthesis at the 3′ terminus.

## 1. Flavivirus

Flaviviruses are important human pathogens that are transmitted by mosquitoes or ticks. Members of flavivirus include dengue (DEN), Zika (ZIK), West Nile (WN), Japanese encephalitis (JE), yellow fever (YF) and tick-borne encephalitis viruses (TBEV), all of which cause wide-spread death and disease throughout the world. For example, dengue virus (DENV) causes diseases ranging from mild dengue fever with non-specific flu-like symptoms to fatal dengue hemorrhagic fever and dengue shock syndrome [1]. The incidence of DENV infection, caused by one of the four serotypes of DENV (DENV1-4), has increased dramatically in recent decades. The CDC estimates that up to 400 million people are infected with DENV; approximately 100 million people show symptoms, and 22,000 people die from severe dengue diseases [2]. Similarly, ZIKV disease, while typically caused by mosquito bites, can spread from a pregnant woman to her fetus, causing microcephaly and other neurological disorders [3]. With the rapid increase in Zika virus transmission, the WHO declared the Zika virus pandemic a public health emergency of international concern in 2016. Despite the significant impact of flavivirus infection on human health and looming threats of future flavivirus epidemics, vaccines are available only for a limited number of flaviviruses, and no antiviral therapies to treat viral infections are available for any flavivirus.

## 2. Flaviviral Genome Structure

The flavivirus genome is an ~11 kb-long, positive-sense, single-stranded RNA (ssRNA), and contains a 5′ untranslated region (5′ UTR), a single open reading frame (ORF), and a 3′ untranslated region (3′ UTR) (Figure 1) [4]. The 5′ terminus of the viral genome is modified by a type 1 cap structure (^m7^GpppN^m^-RNA, where the guanosine cap and first nucleotide of the RNA are methylated), while the 3′ terminus lacks a poly(A) tail. The 5′ UTR spans approximately 100 nt, and the 3′ UTR ranges from 400 to 700 nt in length, depending on the virus species [5]. The 5′ and 3′ UTRs of flavivirus contain several conserved RNA structural motifs that are essential for viral replication and pathogenicity. The 5′ UTR of flavivirus genomes contains two stem-loop structures, stem-loops A and B (SLA and SLB) (Figure 1B). SLA, consisting of the first ~70 nucleotides of the genome, functions as a viral RNA promoter for the viral polymerase NS5 [6,7]. The shorter SLB contains an RNA region called 5′UAR (5′ upstream AUG region) that is complementary to a region in the 3′ UTR (see below) [8]. The 3′ UTR contains several stem-loop structures (SL), one or two dumbbell-like secondary structures (DB1 and DB2), a small hairpin (3′sHP) and a 3′ stem-loop (3′ SL) (Figure 1B). Processing of the stem-loops in the 3′ UTR leads to generation of subgenomic flavivirus RNAs (sfRNAs), which are involved in overall pathogenicity and evasion of the interferon response [9,10,11].

The single ORF is translated into a single polyprotein consisting of ten viral proteins: C-prM-E-NS1-NS2A-NS2B-NS3-NS4A-NS4B-NS5 (Figure 1A). The three structural proteins, capsid (C), pre-membrane (prM), and envelope (E) proteins are involved in the assembly of virions. The C protein forms a nucleocapsid core with the viral RNA genome, and the prM and E proteins assemble into a virus shell that encapsidates the nucleocapsid core. The seven non-structural (NS) proteins, NS1, NS2A/B, NS3, NS4A/B, NS5 are involved in viral genome replication and polyprotein processing. The NS proteins form a viral replication complex on the cytoplasmic side of ER membrane and synthesize multiple copies of viral RNA. Although all viral NS proteins are found in the viral replication complex, only NS3 and NS5 have enzymatic activities required for viral RNA synthesis [12,13] (Figure 2). NS3 consists of an N-terminal protease domain and a C-terminal helicase domain. The NS3 protease requires NS2B as a cofactor, and cleaves the polyprotein from the cytoplasmic side [14,15]. The NS3 helicase has 5′ RNA triphosphatase, nucleoside triphosphatase, and helicase activities, and is involved in the type 1 cap formation at the 5′ terminus of the viral genome [16,17]. NS5 also consists of two domains, an N-terminal methyltransferase and a C-terminal RNA-dependent RNA polymerase (RdRp) domain. NS5 methyltransferase has the RNA guanylyltransferase (GTase) activity, which transfers the GMP cap to the 5′ terminus of viral RNA, and the *N*-7 guanine and 2′-O ribose methyltransferase activities (N7-MTase and 2′O-MTase) that transfer a methyl group to capped RNA to form a type 1 cap structure (Figure 2 inset) [18,19]. The C-terminal polymerase domain is responsible for viral RNA synthesis [20].

## 3. Flavivirus Genome Replication Steps

Flaviviral genome replication steps involve viral RNA synthesis via a negative-strand intermediate and type 1 cap formation at the 5′ end of the newly synthesized positive-strand RNA. First, the viral NS5 polymerase (the C-terminal domain of NS5) uses the genomic positive-sense RNA as a template and synthesizes a complementary negative-sense RNA. NS5 recognizes a conserved RNA stem-loop structure called stem-loop A (SLA) within the 5′ UTR as a promoter, yet initiates negative-strand synthesis at the 3′-end of the genome (Figure 2, step 1) [6]. The newly synthesized, negative-strand remains base paired with the positive strand, resulting in a dsRNA intermediate [21,22]. Next, NS5 polymerase uses the negative strand within the dsRNA as the template to synthesize complementary positive-strand RNA (Figure 2, step 2). The nascent, positive strand displaces the pre-existing positive strand in the dsRNA intermediate. As a result, a positive strand and a new dsRNA intermediate will be produced. The dsRNA intermediate is then recycled to synthesize multiple copies of positive-strand RNA. Thus, RNA synthesis in flavivirus is asymmetric in that the positive-strand RNA is predominantly formed over the negative-strand RNA [22,23]. Please see Section 7 for further discussion.

During viral replication, the positive-strand RNA needs to be modified with a type 1 cap structure (^m7^GpppN^m^-RNA, Figure 2 inset), which requires additions of a GMP cap and methyl groups to the 5′ end of the RNA. RNA capping and methylation likely occur co-transcriptionally during the initial stages of positive-strand RNA synthesis, but little is known about timing or mechanism regarding how flavivirus coordinates RNA synthesis and 5′ end RNA capping [12]. The cap has been shown to be present only on the genomic positive-strand RNA, and not on the dsRNA intermediate in WNV-infected cells [22]. Thus, with the exception of the first cycle, where genomic RNA is used as a template to synthesize negative-strand RNA, the dsRNA intermediate would not contain a 5′ cap in the positive-strand RNA (Figure 2). As in eukaryotic type 1 cap formation, flavivirus requires four sequential enzymatic activities [24]. First, NS3 helicase dephosphorylates the 5′-triphosphate of the positive-strand RNA to diphosphate using its triphosphatase activity (ppp-RNA → ppRNA, Figure 2, step 3). Next, NS5 methyltransferase transfers a GMP moiety from GTP to the 5′-end diphosphate using its guanylyltransferase activity (ppRNA → GpppRNA, Figure 2, step 4) [18]. Then, NS5 methyltransferase methylates the guanosine cap at the N7 position and subsequentially at the ribose 2′-OH position of the first nucleotide (GpppRNA → ^m^GpppRNA → ^m^GpppN^m^-RNA, Figure 2, step 5). NS5 methyltransferase has both N7-MTase and 2′O-MTase activities. The protein uses S-adenosyl methionine (AdoMet) as a methyl donor and releases the byproduct S-adenosyl homocysteine (AdoHcy). The N7 and 2′O methylation reactions require distinct RNA sequences and lengths [25,26]. The N7 cap methylation requires the presence of the ~70 nucleotide-long, stem-loop A in the 5′ UTR of the viral genome, while 2′O methylation requires ~20 nucleotides of the 5′ viral RNA with specific nucleotides at the first and second positions [27].

## 4. Viral RNA Elements Essential for Genome Replication

Historically, the genomic RNA of RNA viruses has been considered to simply code for viral proteins, and thus the information content limited to its primary sequence. However, it has become clear over the past several years that the genomic RNA performs additional functions in replication and immunity that are coded in the 3-dimensional structure of the RNA itself. There are two essential elements in flaviviral RNA genomes that are required for viral RNA synthesis, the SLA at the 5′ UTR and three pairs of complementary circularization sequences at the 5′ and 3′ UTRs (Figure 1B) [8,28,29,30]. The predicted secondary structures of flaviviruses SLAs include a three-way (3-way) junction structure consisting of the top stem-loop, side stem-loop, and bottom stem, which were predicted to assemble an overall structure resembling the letter ‘Y’ (Figure 3A,B) [8]. The viral polymerase NS5 specifically recognizes the SLA as an RNA promoter to initiate negative-strand RNA synthesis beginning at the 3′ end of the viral genome. Consequently, flaviviruses that contain deletions or mutations in the SLA region are replication defective [8,28]. Although the sequence identity between various flavivirus SLAs is relatively low, the predicted 3-way junction and promoter activity of SLA are conserved among all flaviviruses [30]. Further, flavivirus can use an SLA promoter from a related virus for viral replication. For example, an WNV genome containing a DENV2 SLA can replicate as well as wild-type virus [31]. This suggests that flaviviruses share a common promoter structure and conserved mechanism for initiation of replication.

The presence of SLA is necessary for viral genome replication, but not sufficient, and flaviviral genome replication requires long-range RNA–RNA interactions between the 5′ and 3′ termini of the genome [29,30,32]. The first set of circularization sequences is the UAR (upstream AUG region) located within stem-loop B in the 5′ UTR and its complementary sequence 3′-UAR, located within the 3′ SL (Figure 1B). Additional circularization sequences DAR (downstream AUG region) and CS1 (conserved sequence 1) at the 5′ end of viral genome are complementary to the corresponding 3′-DAR and 3′-CS at the 3′ UTR, respectively (Figure 1B). Because 5′ DAR and CS circularization sequences are located in the coding region of the capsid protein, circularization of viral genome would inhibit viral protein translation. Thus, the flaviviral genome is thought to exist in two forms, a linear and a circular form (Figure 1C). The linear form of the genome would be required to initiate viral RNA translation. Following viral protein translation, the viral genome is circularized, mediated by the circularization sequences at the 5′ and 3′-ends of the viral genome. This would bring the 3′ end of the viral genome closer to the SLA at the 5′ UTR [7,33]. Circularization of viral genome using 3′ DAR within the 3′ SL would also change the 3′ terminal nucleotide structure from a stem-loop to an unpaired single strand. The viral polymerase NS5 can then specifically recognize the SLA at the 5′ terminus of the viral genome and initiates negative-strand RNA synthesis from the adjacent single-stranded 3′ end of the circularized viral genome (Figure 1C) [6].

## 5. Structure of Viral RNA Promoter SLA

Recent crystal structures of DENV and ZIKV SLAs show that both SLAs consist of a top stem-loop, a side loop, and a bottom stem (Figure 3). Both SLAs form a letter ‘L’-shaped structure with a different angle between the top and bottom stems of the L [34]. The DENV and ZIKV SLA structures differ in the lengths of the bottom stem and top stem-loop, and their relative orientations (Figure 3C,D). The structures show base pairing patterns near the 3-way junction (where the top stem-loop, side loop, and the bottom stem meet) that differ from their predicted secondary structures. In particular, self-complementary side loop sequences are involved in the intermolecular interactions with the side loop of another SLA molecule, rather than participating in the predicted intramolecular base-pair interaction [34]. Further, it was shown that SLA forms a dimer in solution, consistent with the structure, though the function of dimerization is currently unclear [34].

**Figure 3:** Structure of flavivirus stem-loop A (SLA) promoter. (**A**) Sequence conservation in flavivirus SLAs. A graphical presentation of nucleotide sequences for each position is shown. The overall height of the stack indicates the sequence conservation at that position, and the height of symbols within the stack indicates the relative frequency of each nucleotide. SLA sequences of DENV1-4 (NCBI accession numbers, NC_001477, NC_001474, NC_001475, NC_002640), WNV (NC_001563), JEV (NC_001437), and ZIKV (KU527068) were used in the alignment. The figure is generated by WebLogo [35]. (**B**) The predicted secondary structure of DENV2 SLA. The secondary structure was predicted by the program RNAfold [36]. (**C**) The crystal structure of DENV2 SLA. Flavivirus SLA consists of a top stem-loop (red), a side loop (green), and a bottom stem (blue). The positions of the U-bulge and AG motif were indicated. The secondary structure based on the tertiary structure is shown on the right. (**D**) The crystal structure of ZIKV SLA. The crystal structure of ZIKV SLA and its secondary structure are shown. ZIKV SLA is colored as in (**C**).

Mutational studies have identified nucleotides in SLA that are important for viral replication. The U-bulge (at least one unpaired U) in the bottom stem and the ‘AG’ sequence in the apical loop of the top stem-loop were shown to be essential for viral replication [8,33]. Both the U-bulge and the AG-loop sequences are highly conserved in flavivirus SLAs (Figure 3A). When the structures of DENV and ZIKV SLAs are superposed by the highly conserved bottom stem, the U-bulges in both structures are located in the same position, while the AG-loop is related by an ~180° rotation (see below). Additionally, formation of base pairs in the bottom stem, the length of the top stem, and the presence of side loop are required for optimal viral replication [6,8,37]. Interestingly, many mutations that impair viral replication do not prevent NS5-SLA interactions. Even mutations in the AG motif in the top stem-loop, which abolished viral replication, had an identical NS5 binding affinity of ~10 nM [33]. These experiments suggest that NS5 recognizes the overall shape of SLA with few nucleotide-specific interactions with SLA structures [28]. The studies also suggest that SLA recognition by viral polymerase alone is not sufficient for efficient viral replication.

## 6. SLA Promoter-Mediated Negative-Strand RNA Synthesis

DENV2 containing the ZIKV SLA is shown to replicate as well as the wild-type DENV2, suggesting that DENV2 NS5 polymerase can recognize both DENV2 and ZIKV SLA as a promoter to initiate RNA synthesis [36]. This raises a question—how can DENV2 NS5 recognize the two different conformations adopted by DENV and ZIKV SLA? In the absence of the structure of the NS5-SLA complex, it is not clear how NS5 engages the SLA promoter. NS5 consists of an N-terminal MTase and a C-terminal RdRp domain, and structures of NS5 show two major arrangements of RdRp domain relative to the MTase domain (Figure 4A), suggesting that NS5 may accommodate the two different SLA structures by rearranging the relative orientations of the two domains. During viral genome replication, NS5 interacts with SLA at least twice for separate RdRp and MTase functions. NS5 recognizes SLA as an RNA promoter to initiate negative-strand RNA synthesis (RdRp function) [6]. NS5 also recognizes SLA as the substrate for 5′ cap methylation at the N7 position (MTase function) [27]. In this case, the 5′ cap covalently linked to the bottom stem of SLA would be positioned in the MTase active site. Fluorescence-based SLA binding assays identified that SLA binds to both the MTase and the RdRp domains of NS5, and that the SLA-binding site does not overlap with the template-binding channel of RdRp [28,38]. This result indicates that SLA and ssRNA template can bind NS5 simultaneously. Additionally, mutations of R22-K23 in the MTase and K841-R842 in the thumb subdomain of RdRp reduce SLA binding affinity by 2-3 fold. The NS5 RdRp and SLA interaction via the thumb subdomain of RdRp was also suggested by a refined yeast three-hybrid scan [39]. Thus, a model of the NS5 and SLA complex, wherein the 5′ terminus of SLA binds the MTase active site and the top stem-loop binds in the thumb subdomain of RdRp was proposed [34]. This model allows the 3′ end of viral genome to concomitantly bind to the template-binding channel of NS5 without the need of additional conformational change to accommodate the 3′ end of the genome following genome cyclization (Figure 1C and Figure 4B). In this model, NS5 recognizes the large SLA via the high-affinity SLA-binding site and recruits the 3′-end of viral genome near the template-binding channel [36]. The 3′-end of viral genome, positioned in the RdRp active site, will then be copied by de novo RNA synthesis [19]. The model suggests that SLA remains bound to NS5 during elongation until it is time for the SLA at the 5′-end to become the template at the very end of replication. This prolonged NS5 and SLA interaction would accomplish selective viral RNA synthesis during genome replication. By recognizing both the 5′ end SLA and the 3′ end of the viral genome, flavivirus can sequester only intact viral RNAs on NS5, avoiding the myriad of cellular RNAs in the cytoplasm, thus ensuring that the viral polymerase copies only complete viral genomes that include both the SLA at the 5′-end and the 3′ terminus.

## 7. Positive-Strand RNA Synthesis

NS5 catalyzes both negative- and positive-strand RNA synthesis. During virus replication, 10-50-fold higher amounts of positive-strand RNA are synthesized compared to negative-strand RNA [23], and thus NS5 polymerase spends the majority of its time synthesizing positive-strands from the dsRNA intermediate (Figure 2). However, the mechanism of positive-strand RNA synthesis is not well understood. The requirements of positive- and negative-strand synthesis are different regarding their templates (dsRNA for positive-strand synthesis vs. genomic ssRNA for negative-strand synthesis), products (positive-sense ssRNA vs. dsRNA), and downstream modifications (type 1 cap formation for positive strand vs. no modification for negative strand). It is currently not known how NS5 recognizes negative strand as a template in the context of a dsRNA intermediate. During positive-strand RNA synthesis, the dsRNA intermediate must be separated into two strands, and the 3′ terminus of the negative strand enters the polymerase active site. This step is poorly understood due to a paucity of structural information regarding the genomic RNA and the lack of an in vitro viral replication assay. Although it was assumed that viral helicase NS3 would unwind the dsRNA during positive-strand RNA synthesis, NS3 is unable to separate blunt-ended dsRNA [40,41]. Thus, NS3 helicase is unlikely to be involved in its initial separation. Alternatively, it is possible that the termini of the dsRNA intermediate are not completely annealed and may be separated via thermal fluctuations [42]. This process may be facilitated by the formation of stable stem loops of SLA at the 5′ end of the viral genome and its complementary structure at the 3′ end of the negative-strand that we refer SLA(-).

The identity of the promoter for positive-strand RNA synthesis is also unclear. Following separation of the dsRNA intermediate, both SLA and its complementary SLA(-) are exposed in the positive and negative strand, respectively. It is not clear whether NS5 binds to SLA or SLA(-) to synthesize positive-strand RNA. Currently, there is no widely accepted mechanism for positive-strand RNA synthesis in flavivirus, and biochemical data exist to support both SLA and SLA(-) as the promoters for positive-strand synthesis. For example, WNV NS5 is able to use the 3′-terminal 230 nt of the negative-strand to synthesize RNA [43]. This template contains SLA(-), and thus WNV SLA(-) may function as a promoter and interact with NS5 to initiate positive-strand RNA synthesis. Additionally, DENV SLA in the positive-strand RNA can also function as a promoter to synthesize RNA *in trans* [8,20]. For example, DENV2 NS5 cannot synthesize RNA from the 3′-terminal 373 nt of positive-strand [20]. However, when the template is annealed with the complementary, 5′-terminal positive-strand (which contains SLA), NS5 can synthesize RNA from the 3′ end of each template [20]. This result suggests that DENV SLA in the positive-strand RNA can functions as the promoter to synthesize positive-strand RNA.

## 8. Conclusions and Perspectives

The identification of SLA as an RNA promoter for flavivirus polymerase NS5, and the structural studies of the SLA promoter and NS5 have provided insight into how flavivirus selectively replicate the viral genome using specific interactions between SLA and NS5. Future studies will be geared toward understanding how the NS5-SLA complex carries out individual steps of RNA replication involving both negative- and positive-strand RNA synthesis, and how the complex coordinates positive RNA synthesis and type 1 cap formation. Future studies on the structure and function SLA(-) would also be needed to determine whether SLA(-) has a role in viral replication.

## Figures and Tables

**Figure 1:** Flavivirus genome organization. (**A**) Genome organization of flaviviruses. The viral genome contains a single open-reading frame (ORF) and is translated into a single polyprotein consisting of structural (C, prM, and E), and the non-structural proteins (NS1, NS2A/B, NS3, NS4A/B, and NS5). The known functions of the viral proteins are listed below. The viral genome is flanked by 5′ and 3′ untranslated regions (UTRs) containing RNA structures important for viral replication. The 5′ terminus of the genome is modified with a type 1 cap structure. (**B**) Flavivirus RNA regions required for viral genome replication. The 5′ UTR consists of two stem-loops, A and B. Stem-loop A (SLA) functions as a viral RNA promoter. The 3′ UTR also consists of several stem-loops (SL), dumb-bell structures (DB1, 2), 3′ small hairpin (3′sHP), and 3′ stem-loop (3′ SL). The genome also contains three complementary sequences in the 5′ and 3′ RNA regions, UAR (upstream AUG region), DAR (downstream AUG region), and CS (conserved sequence). Complementary interactions between the 5′ and 3′ regions facilitate circularization of the viral genome, indicated by red and blue lines. (**C**) Proposed model of flaviviral genome. Flavivirus genome is suggested to exist in a linear form that is required for viral protein translation and in a circular form that is required for viral genome replication [6].

**Figure 2:** Viral RNA synthesis. Both negative-strand (red) and positive-strand (blue) RNA synthesis are carried out by viral polymerase NS5. First, NS5 synthesizes negative-strand RNA using the genomic positive-strand as a template, resulting in dsRNA intermediate (step 1). The close circle indicates the type 1 cap at the 5′ end. NS5 then uses the negative-strand of the dsRNA as a template and synthesizes positive-strand RNA, resulting in a single-stranded positive-sense RNA and a dsRNA intermediate (step 2). For capping and methylations, NS3 dephosphorylates the triphosphate at the 5′ end of positive-strand RNA to diphosphate (step 3). NS5 next transfers a GMP cap from GTP to the 5′ diphosphorylated RNA to form a 5′ to 5′ triphosphate bridge (step 4). NS5 sequentially methylates the guanosine cap at the N7 position and the first nucleotide of viral RNA at the 2′O position using the cofactor S-adenosyl methionine (step 5). The structure of the type 1 cap at the 5′ end of RNA genome is shown in inset.

**Figure 4:** Model of the NS5-SLA complex. (**A**) Domain arrangements in flavivirus NS5 and stem-loop A (SLA). The structures of the flavivirus NS5 and SLA show different relative orientations of their domains. ZIKV and DENV NS5 structures are superposed by their MTase domains; domains are indicated only in DENV NS5 for clarity (left). The ZIKV and DENV SLA structures are superposed by their bottom stems, and the top stem-loop and bottom stem are indicated in DENV SLA (right). (**B**) Model of the NS5-SLA complex. The NS5-SLA complex is modeled based on the binding assays of mutant NS5 and previous biochemical assays. The schematic of SLA interaction with NS5 is shown on the right. The model suggests that flavivirus NS5 recognizes both the 5′ end SLA and the 3′ end of the viral genome, and thus can sequester intact viral RNAs on NS5 to ensure that viral polymerase copies complete viral genomes.

## References

[1] Clyde K., Kyle J.L., Harris E. (2006). Recent advances in deciphering viral and host determinants of dengue virus replication and pathogenesis. J. Virol..

[2] Murray N.E., Quam M.B., Wilder-Smith A. (2013). Epidemiology of dengue: Past, present and future prospects. Clin. Epidemiol..

[3] Miner J.J., Cao B., Govero J., Smith A.M., Fernandez E., Cabrera O.H., Garber C., Noll M., Klein R.S., Noguchi K.K. (2016). Zika Virus Infection during Pregnancy in Mice Causes Placental Damage and Fetal Demise. Cell.

[4] Lindenbach B.D., Thiel H.J., Rice C.M. (2007). Flaviviridae: The Viruses and Their Replication.

[5] Ng W.C., Soto-Acosta R., Bradrick S.S., Garcia-Blanco M.A., Ooi E.E. (2017). The 5′ and 3′ Untranslated Regions of the Flaviviral Genome. Viruses.

[6] Filomatori C.V., Lodeiro M.F., Alvarez D.E., Samsa M.M., Pietrasanta L., Gamarnik A.V. (2006). A 5′ RNA element promotes dengue virus RNA synthesis on a circular genome. Genes Dev..

[7] Gebhard L.G., Filomatori C.V., Gamarnik A.V. (2011). Functional RNA elements in the dengue virus genome. Viruses.

[8] Lodeiro M.F., Filomatori C.V., Gamarnik A.V. (2009). Structural and functional studies of the promoter element for dengue virus RNA replication. J. Virol..

[9] Pijlman G.P., Funk A., Kondratieva N., Leung J., Torres S., van der Aa L., Liu W.J., Palmenberg A.C., Shi P.Y., Hall R.A. (2008). A highly structured, nuclease-resistant, noncoding RNA produced by flaviviruses is required for pathogenicity. Cell Host Microbe.

[10] Slonchak A., Khromykh A.A. (2018). Subgenomic flaviviral RNAs: What do we know after the first decade of research. Antivir. Res..

[11] Chapman E.G., Costantino D.A., Rabe J.L., Moon S.L., Wilusz J., Nix J.C., Kieft J.S. (2014). The structural basis of pathogenic subgenomic flavivirus RNA (sfRNA) production. Science.

[12] Klema V.J., Padmanabhan R., Choi K.H. (2015). Flaviviral Replication Complex: Coordination between RNA Synthesis and 5′-RNA Capping. Viruses.

[13] Welsch S., Miller S., Romero-Brey I., Merz A., Bleck C.K., Walther P., Fuller S.D., Antony C., Krijnse-Locker J., Bartenschlager R. (2009). Composition and three-dimensional architecture of the dengue virus replication and assembly sites. Cell Host Microbe.

[14] Chambers T.J., Grakoui A., Rice C.M. (1991). Processing of the yellow fever virus nonstructural polyprotein: A catalytically active NS3 proteinase domain and NS2B are required for cleavages at dibasic sites. J. Virol..

[15] Falgout B., Pethel M., Zhang Y.M., Lai C.J. (1991). Both nonstructural proteins NS2B and NS3 are required for the proteolytic processing of dengue virus nonstructural proteins. J. Virol..

[16] Li H., Clum S., You S., Ebner K.E., Padmanabhan R. (1999). The serine protease and RNA-stimulated nucleoside triphosphatase and RNA helicase functional domains of dengue virus type 2 NS3 converge within a region of 20 amino acids. J. Virol..

[17] Benarroch D., Selisko B., Locatelli G.A., Maga G., Romette J.L., Canard B. (2004). The RNA helicase, nucleotide 5′-triphosphatase, and RNA 5′-triphosphatase activities of Dengue virus protein NS3 are Mg2+-dependent and require a functional Walker B motif in the helicase catalytic core. Virology.

[18] Issur M., Geiss B.J., Bougie I., Picard-Jean F., Despins S., Mayette J., Hobdey S.E., Bisaillon M. (2009). The flavivirus NS5 protein is a true RNA guanylyltransferase that catalyzes a two-step reaction to form the RNA cap structure. RNA.

[19] Ackermann M., Padmanabhan R. (2001). De novo synthesis of RNA by the dengue virus RNA-dependent RNA polymerase exhibits temperature dependence at the initiation but not elongation phase. J. Biol. Chem..

[20] You S., Padmanabhan R. (1999). A novel in vitro replication system for Dengue virus. Initiation of RNA synthesis at the 3′-end of exogenous viral RNA templates requires 5′- and 3′-terminal complementary sequence motifs of the viral RNA. J. Biol. Chem..

[21] Padmanabhan R., Takhampunya R., Teramoto T., Choi K.H. (2015). Flavivirus RNA synthesis in vitro. Methods.

[22] Wengler G., Wengler G., Gross H.J. (1978). Studies on virus-specific nucleic acids synthesized in vertebrate and mosquito cells infected with flaviviruses. Virology.

[23] Gullberg R.C., Jordan Steel J., Moon S.L., Soltani E., Geiss B.J. (2015). Oxidative stress influences positive strand RNA virus genome synthesis and capping. Virology.

[24] Dong H., Zhang B., Shi P.Y. (2008). Flavivirus methyltransferase: A novel antiviral target. Antivir. Res.

[25] Egloff M.P., Benarroch D., Selisko B., Romette J.L., Canard B. (2002). An RNA cap (nucleoside-2′-O-)-methyltransferase in the flavivirus RNA polymerase NS5: Crystal structure and functional characterization. EMBO J..

[26] Ray D., Shah A., Tilgner M., Guo Y., Zhao Y., Dong H., Deas T.S., Zhou Y., Li H., Shi P.Y. (2006). West Nile virus 5′-cap structure is formed by sequential guanine N-7 and ribose 2′-O methylations by nonstructural protein 5. J. Virol..

[27] Dong H., Ray D., Ren S., Zhang B., Puig-Basagoiti F., Takagi Y., Ho C.K., Li H., Shi P.Y. (2007). Distinct RNA elements confer specificity to flavivirus RNA cap methylation events. J. Virol..

[28] Bujalowski P.J., Bujalowski W., Choi K.H. (2017). Interactions between the Dengue Virus Polymerase NS5 and Stem-Loop A. J. Virol..

[29] Khromykh A.A., Meka H., Guyatt K.J., Westaway E.G. (2001). Essential role of cyclization sequences in flavivirus RNA replication. J. Virol..

[30] Villordo S.M., Gamarnik A.V. (2009). Genome cyclization as strategy for flavivirus RNA replication. Virus Res..

[31] Yu L., Nomaguchi M., Padmanabhan R., Markoff L. (2008). Specific requirements for elements of the 5′ and 3′ terminal regions in flavivirus RNA synthesis and viral replication. Virology.

[32] Friebe P., Harris E. (2010). Interplay of RNA elements in the dengue virus 5′ and 3′ ends required for viral RNA replication. J. Virol..

[33] Filomatori C.V., Iglesias N.G., Villordo S.M., Alvarez D.E., Gamarnik A.V. (2011). RNA sequences and structures required for the recruitment and activity of the dengue virus polymerase. J. Biol. Chem..

[34] Lee E., Bujalowski P.J., Teramoto T., Gottipati K., Scott S.D., Padmanabhan R., Choi K.H. (2021). Structures of flavivirus RNA promoters suggest two binding modes with NS5 polymerase. Nat. Commun..

[35] Crooks G.E., Hon G., Chandonia J.M., Brenner S.E. (2004). WebLogo: A sequence logo generator. Genome Res..

[36] Zuker M., Stiegler P. (1981). Optimal computer folding of large RNA sequences using thermodynamics and auxiliary information. Nucleic Acids Res..

[37] Li X.F., Jiang T., Yu X.D., Deng Y.Q., Zhao H., Zhu Q.Y., Qin E.D., Qin C.F. (2010). RNA elements within the 5′ untranslated region of the West Nile virus genome are critical for RNA synthesis and virus replication. J. Gen. Virol.

[38] Bujalowski P.J., Bujalowski W., Choi K.H. (2020). Identification of the viral RNA promoter stem loop A (SLA)-binding site on Zika virus polymerase NS5. Sci. Rep..

[39] Hodge K., Tunghirun C., Kamkaew M., Limjindaporn T., Yenchitsomanus P.T., Chimnaronk S. (2016). Identification of a Conserved RNA-dependent RNA Polymerase (RdRp)-RNA Interface Required for Flaviviral Replication. J. Biol. Chem..

[40] Zhong W., Ingravallo P., Wright-Minogue J., Skelton A., Uss A.S., Chase R., Yao N., Lau J.Y., Hong Z. (1999). Nucleoside triphosphatase and RNA helicase activities associated with GB virus B nonstructural protein 3. Virology.

[41] Huang Z.S., Wang C.C., Wu H.N. (2010). HCV NS3 protein helicase domain assists RNA structure conversion. FEBS Lett..

[42] Ertel K.J., Brunner J.E., Semler B.L. (2010). Mechanistic consequences of hnRNP C binding to both RNA termini of poliovirus negative-strand RNA intermediates. J. Virol..

[43] Nomaguchi M., Teramoto T., Yu L., Markoff L., Padmanabhan R. (2004). Requirements for West Nile virus (−)- and (+)-strand subgenomic RNA synthesis in vitro by the viral RNA-dependent RNA polymerase expressed in Escherichia coli. J. Biol. Chem..

